The article "Investigation of the Mechanism of Periploca forrestii against Rheumatoid Arthritis with Network Pharmacology-Based Analysis" was published in 2022. Journal: Evid Based Complement Alternat Med.

# Investigation of the Mechanism of *Periploca forrestii* against Rheumatoid Arthritis with Network Pharmacology-Based Analysis

**DOI:** 10.1155/2022/2993374

**Published:** 2022-07-05

**Authors:** Qiuyi Wang, Xueming Yao, Yi Ling, Ying Huang, Changming Chen, Lei Hou, Yutao Yang, Hongyan Wu, Wukai Ma

**Affiliations:** ^1^Clinical Medical College, Jiangxi University of Traditional Chinese Medicine, Nanchang 330000, China; ^2^Department of Rheumatology and Immunology, The Second Affiliated Hospital of Guizhou University of Traditional Chinese Medicine, Guiyang 550001, China; ^3^Shenzhen Luohu District Hospital of Traditional Chinese Medicine, Shenzhen 518001, China

## Abstract

*Periploca forrestii* Schltr (*P. forrestii*) is an edible medicinal herb with various health benefits such as treating antirheumatoid arthritis (RA), reducing inflammation, and preventing tumor growth. The active ingredients in *P. forrestii* responsible for its protective effect against RA, however, remain unknown. In this study, the active ingredient of *P. forrestii* and its potential mechanism of action against RA were investigated by network pharmacology and enrichment analysis. The methods included predicting target genes of P. forrestii, constructing a protein interaction network, and performing gene-ontology (GO) and Kyoto-encyclopedia of genes and genomes (KEGG) enrichment analysis. We discovered targets of RA through retrieval of OMIM and GeneCards public databases. Cardiac glycosides (CGs) are considered the primarily active ingredients of *P. forrestii*, and the target genes of GCs were discovered to be overlapped with relevant targets of RA using the Venn diagram. After that, prediction of relevant targets of P. forrestii was accomplished with a network pharmacology-based approach. Through the Venn diagram, we discovered 99 genes shared in the target genes of *P. forrestii* and RA. Gene enrichment analysis showed that the mechanisms of CGs against RA are associated with 55 signaling pathways, including endocrine resistance, Epstein-Barr virus infection, bladder cancer, prostate cancer, and coronavirus disease (COVID-19) signaling pathways. Coexpression analysis indicated ADSL, ATIC, AR, CCND1, MDM2, and HSP90AA1 as the hub genes between putative targets of *P. forrestii*-derived CGs and known therapeutic targets of RA. In conclusion, we clarified the mechanism of action of *P. forrestii* against RA, which would provide a basis for further understanding the clinical application of *P. forrestii.*

## 1. Introduction

Rheumatoid arthritis (RA), one of the most common auto-immune diseases, is characterized by the destruction of articular cartilage (AC), synovial hyperplasia, and pannus formation [1]. RA also ranks among the top ten causes of disability worldwide. It has been shown that people with RA are considerably burdened by irreversible deformities and even dysfunction of the joints, which adversely affect the quality of life of these individuals [1]. However, the development of effective prophylactic and therapeutic treatments has been hampered by the complexity of RA's etiology as well as the lack of clarity on its pathogenesis, which is thought to involve both genetic and environmental components [2–4] identifying as anticancer, antidiarrheal, antidepressant, anti-inflammatory, analgesic, and thrombolytic agents [5–10]. RA is a complex disorder, and due to the various properties, a variety of TCMs have played a vital role in controlling RA symptoms, thus assisting anti-RA and nonsteroidal anti-inflammatory drugs [11–14].

The article "Investigation of the Mechanism of Periploca forrestii against Rheumatoid Arthritis with Network Pharmacology-Based Analysis" was published in 2022. Journal: Evid Based Complement Alternat Med.

*Periploca forrestii* Schltr (*P. forrestii*, also known as *Hei-Long-Gu* or *Hei-Gu-Teng*) is derived from the rhizomes and roots of a vining shrub of Periploca (Asclepiadaceae). For thousands of years, *P. forrestii* has been regarded as one of the most widely used Chinese herbal medicines (CHM) in Guizhou, China. It is historically believed to possess numerous medicinal properties, including activating the meridians, improving blood circulation, dispelling wind, and removing dampness, as well as being used to treat RA, bruises, and tumors [15]. Until now, the increased interest in CHM has led researchers to isolate and identify over 100 active compounds from *P. forrestii*. This means that CHM, *P. forrestii*, and its periplocin derivatives can exert anti-inflammatory activity by regulating the immune response. For example, in rats with adjuvant arthritis (AIA), *P. forrestii* has been shown to inhibit local joint inflammation and bone destruction [16]. Additionally, studies in pharmacology have indicated that cardiac glycosides (CGs) are the major active ingredients of *P. forrestii* which have wound healing and antitumor properties [17–19]. Despite the fact that *P. forrestii* has been extensively investigated for its therapeutic use in a variety of human diseases, our knowledge of its mechanism of action in treating RA is still restricted. Therefore, this study was undertaken in order to investigate the possible mechanisms of action of *P. forrestii*-derived CGs when these compounds are applied in RA treatment.

## 2. Materials and Methods

### 2.1. Chemical Structure of Compounds

Firstly, based on literature mining, we gathered information on the main active ingredients of *P. forrestii*-derived CGs. Next, the chemical structures of these gathered active ingredients were retrieved from the PubChem database. As an open-archive, the PubChem database (https://pubchem.ncbi.nlm.nih.gov/) consists of compound, substance, and bioassay primary databases.

The article "Investigation of the Mechanism of Periploca forrestii against Rheumatoid Arthritis with Network Pharmacology-Based Analysis" was published in 2022. Journal: Evid Based Complement Alternat Med.

### 2.2. Prediction of CGs Targets

Through the use of the pharmacophore mapping approach (PMA), we were able to identify potential therapeutic targets for these retrieved compounds in the PharmMapper (PM) database (http://www.lilab-ecust.cn/pharmmapper/) [20–22]. After that, the 3D chemical structures of these compounds were inputted into the PM database, and then twenty human targets with the highest matching scores were chosen for each of the compounds. Also, we removed probable CGs-related predicted targets that were repeated or nonstandard.

### 2.3. Analysis of Protein-Protein Interaction Network (PPIN) and Visualization

For predicted drug targets and known RA-related targets, an interaction network was selected with a score greater than or equal to 0.4 for the construction of a PPI network in a database, the Search Tool for Retrieving Interactive Genes (STRING). In light of the built interaction network, using the R package, we identified adjacent nodes with a greater number of connections to other nodes in our networks. For the purpose of constructing and visualizing interaction networks, Cytoscape software (Version 3.9.0) was used. The network displayed the active ingredients of CGs, and the nodes on the periphery of the network represented the key target genes of diseases and active components of CGs. As a result, the entire network demonstrates the link between drug-bioactive components-disease targets, while the mechanistic action of *P. forrestii* in RA treatment was explored by constructing this network.

### 2.4. SIN Targets Prediction for Treatment of RA

By searching for the term “rheumatoid arthritis” in the databases of GeneCards (https://www.genecards.org/) [23] and OMIM (https://www.omim.org/) [24], it was possible to retrieve therapeutic targets associated with RA. Moreover, using the Venn diagram, we were able to identify the overlapping genes between putative targets of *P. forrestii* and known therapeutic targets of RA.

### 2.5. Enrichment Analysis of Gene-Ontology (GO) and Kyoto-Encyclopedia of Genes and Genomes (KEGG) Pathway

A GO functional annotation was performed using the org.Hs.eg.db R package, while principal target genes of *P. forrestii* in RA treatment were converted into EntrezID for GO function enrichment analysis of the aforementioned genes (*p* < 0.05). Subsequently, we discovered key signaling pathways with overlapping targets and biological functions through KEGG pathway analysis, wherein *p* < 0.05.

## 3. Results

### 3.1. Target Genes that Associated with 10 Compounds and RA

As a result of a literature review, the 10 main chemical components of CGs obtained from *P. forrestii* were collected, and 654 corresponding target genes were determined using the pharmacophore model prediction tool. Afterward, we summarized and deduplicated the data in order to obtain 10 species with 279 target genes corresponding to the 10 main chemical components. Through GeneCards and the OMIM database, a total of 4821 target genes relating to RA were obtained. We performed a Venn diagram analysis on the target genes of CHM components and RA, resulting in 99 intersecting genes (Figure 1).

The article "Investigation of the Mechanism of Periploca forrestii against Rheumatoid Arthritis with Network Pharmacology-Based Analysis" was published in 2022. Journal: Evid Based Complement Alternat Med.

### 3.2. Potential Signaling Pathways of CGs against RA

Based on these identified target genes, an analysis on a total of 29 GO term lists that were related to RA was performed (Figures 2(a) and 2(b)). These lists were combined with the top 20 results from a gene enrichment analysis of targets. As a result, this GO enrichment analysis showed biological processes and functions related to the activity of ligand activated transcription factors, the activity of nuclear-receptor, Hsp90 protein-binding, ubiquitin-like protein ligase-binding, RNA polymerase-II transcription initiation factor-binding, and so forth. There were also 55 signaling pathways that were identified in the KEGG analysis of *P. forrestii* (*p* < 0.05). Taken together, *P. forrestii* may treat RA by influencing endocrine resistance, Epstein-Barr virus infection, bladder cancer, prostate cancer, and COVID-19 signaling pathways, as well as other pathways (Figures 2(c) and 2(d).  Table 1).

### 3.3. Hub Genes of CGs against RA

We used the online STRING database to construct a protein-protein interaction (PPI) network of overlapped targets with 4722 RA-related genes and 180 CGs-related genes (Figure 3(a)). Before it was used to visualize the overlapping genes between CGs and RA, the PPI network was constructed utilizing the STRING database and Cytoscape.

### 3.4. Construction of Coexpression Network

Within the PPI network, the circle denotes the size of the degree value; a higher degree value corresponds to a transition from the color red to the color blue. The thickness of the edge represented the size of the combined score; a thicker edge suggests that the combined score has a bigger value. ADSL, ATIC, AR, CCND1, MDM2, and HSP90AA1 were among the key protein nodes, which were produced based on the credit scores of node interactions (Figure 4).

## 4. Discussion

As a result of their chemical diversity and advantages such as simple availability and bioprocessing, scientists have always been interested in natural compounds [25–27]. *P. forrestii* has been reported to contain numerous bioactive compounds, including steroids, flavonoids, and phenylpropanoids [25]. These active molecules have previously shown a variety of functions, including antiproliferative, antioxidant, antinociceptive, and palliative effects [28–33]. In addition, TCMs containing these bioactive compounds have been demonstrated to be effective against COVID-19, showing their antivirus properties [34]. No doubt, *P. forrestii* and its extracts are capable of exhibiting these similar properties. Among the identified compounds in *P. forrestii* extracts, CGs are considered to be the main bioactive component. The CGs are mainly obtained from various plant and amphibian sources, such as members of the genus Bufo [35, 36]. It is widely accepted that heart disease and cancer treatment can benefit greatly from the application of these GCs, with some undergoing clinical trials (phase I and II) for solid tumor therapy [37–39].

The article "Investigation of the Mechanism of Periploca forrestii against Rheumatoid Arthritis with Network Pharmacology-Based Analysis" was published in 2022. Journal: Evid Based Complement Alternat Med.

In this study, the pharmacophore model was used to predict active compounds of CGs, and a network of “drug-active ingredient-disease” was built, in which we attempted an analysis of the CGs' mechanism of action. Besides, a coexpression network was established using the STRING database and used to identify key target genes. Furthermore, we performed function analysis of GO and KEGG pathway to reveal the related signaling pathways.

In light of our findings, enrichment analysis indicated that the treatment of RA with *P. forrestii* may be related to endocrine resistance, Epstein-Barr virus infection, bladder cancer, prostate cancer, and COVID-19 signaling pathways, suggesting that *P. forrestii* might treat RA by altering these signaling pathways. There is a long-established association between RA and cancer, based on studies that have demonstrated an increased lymphoma risk in patients with RA [40]. Though not all types of cancer are equally at risk, lung cancer and lymphoma incidences are higher among RA patients than in the general population as demonstrated by standardized incidence rates [41]. Therefore, CGs participate in a wide range of cancer-related pathways that are involved in RA treatment, which provides a novel perspective for the combination therapy. Not just cancer, but also COVID-19 was discovered to be connected with RA. According to the findings of Williamson and colleagues [42], people with RA, systemic lupus erythematosus, or psoriasis (combined) were more likely to die of COVID-19. Other researchers have also observed that some common treatment strategies like cytokine inhibition were effective in both COVID-19 and RA [43]. Furthermore, it was found that analysis of the GO function enrichment of core genes was primarily concentrated in the activity of ligand activated transcription factor, nuclear-receptor, Hsp90 protein-binding, ubiquitin-like protein ligase-binding, and RNA polymerase-II transcription initiation factor-binding. However, the current research on *P. forrestii* did not report on this specific aspect, which needs further investigation. Likewise, our coexpression analysis revealed that ADSL, ATIC, AR, CCND1, MDM2, and HSP90AA1 were the key genes that linked potential targets of *P. forrestii* to known therapeutic targets within RA.

The article "Investigation of the Mechanism of Periploca forrestii against Rheumatoid Arthritis with Network Pharmacology-Based Analysis" was published in 2022. Journal: Evid Based Complement Alternat Med.

Through these molecular mechanisms, CGs may play an important role in treating RA, thereby providing a theoretical foundation for future research and clinical application of these organic compounds. Also, based on their antitumor property, GCs have been increasingly studied, exhibiting cytotoxic effects against some tumor types, including prostate cancer [44, 45], melanoma [37], and lung cancer [46–48]. In view of this, the CGs' potential mechanism and potential *in vivo* application deserve further study. On the other hand, although CGs have shown some excellent safety profiles and efficacy, future clinical trials will need to confirm the long-term efficacy and safety of their extracts and chemical components due to the complexity of *P. forrestii* compounds.

## 5. Conclusion

In summary, a network of essential genes was established using the network pharmacology-based approach, connecting the putative therapeutic targets of *P. forrestii* to the known targets of RA. This network screened out six hub genes, including ADSL, ATIC, AR, CCND1, MDM2, and HSP90AA1. The significant biological processes, molecular functions, cellular components, and KEGG pathways were obtained by performing GO and KEGG pathway analysis. The hub genes and enrichment analysis results indicated that the primary active ingredients, GCs, appeared frequently in the application to treat RA, cancer, and COVID-19. The therapeutic effect of GCs in treating RA is mainly by regulating ligand activated transcription factors, activity of nuclear-receptor, Hsp90 protein-binding, ubiquitin-like protein ligase-binding, and RNA polymerase-II transcription initiation factor-binding. These pathways were most commonly observed in the host's immune inflammatory response, oxidative stress, cell repair, and cell migration. These findings provide a basis for understanding the further clinical application of *P. forrestii* and its ingredients, GCs, in the treatment of RA.

## Figures and Tables

**Figure 1:** Using a Venn diagram analysis, 4722 target genes for the CHM component, GC, as well as 180 target genes for rheumatoid arthritis were identified, resulting in 99 overlapping genes.

The article "Investigation of the Mechanism of Periploca forrestii against Rheumatoid Arthritis with Network Pharmacology-Based Analysis" was published in 2022. Journal: Evid Based Complement Alternat Med.

**Figure 2:** The top 20 gene-ontology (GO) categories of overlapping genes between RA and cardiac glycosides (CGs) were presented in a histogram and bubble diagram, respectively (a, b). The top 20 KEGG signaling pathways of overlapping genes were presented in a histogram and bubble diagram, respectively (c, d).

**Figure 3:** Key gene nodes in the rheumatic arthritis (RA)-related gene protein network (a). The interaction network of cardiac glycosides (CGs) and disease-related genes (b). Among them, the green diamonds represent the active components of CGs, whereas the pink circles represent key target genes, and the pink lines denote the relationship between each target gene.

**Figure 4:** Coexpression network of related genes and target proteins.

**Table 1:** Top 10 target genes related to the occurrence and development of rheumatoid arthritis (RA) revealed by enrichment set analysis.

Pathway ID	Description	Gene ID	p.adjust
hsa01522	Endocrine resistance	MMP2/NOTCH1/HBEGF/E2F1/MAPK9/ESR1/ERBB2/CCND1/MDM2/ESR2	6.83E-06
hsa05169	Epstein-barr virus infection	B2M/CDK2/BTK/RAC1/E2F1/MAPK9/Table1/CCND1/IKBKG/EIF2AK2/MDM2/IRAK4	5.51E-05
hsa05219	Bladder cancer	MMP2/HBEGF/E2F1/ERBB2/CCND1/MDM2	1.83E-04
hsa05215	Prostate cancer	CDK2/E2F1/ERBB2/CCND1/AR/IKBKG/MDM2/HSP90AA1	2.30E-04
hsa05171	Coronavirus disease-COVID-19	F13A1/C2/HBEGF/F2/MAPK9/IKBKG/EIF2AK2/IRAK4/FCGR2A/RPS3/IL6ST	6.10E-04
hsa05167	Kaposi sarcoma-associated herpesvirus infection	IFNGR1/MAPKAPK2/HCK/RAC1/E2F1/MAPK9/CCND1/IKBKG/EIF2AK2/IL6ST	6.30E-04
hsa05203	Viral carcinogenesis	CDK2/MAPKAPK2/RAC1/CCND1/DDB1/IKBKG/EIF2AK2/MDM2/HDAC6/IL6ST	7.63E-04
hsa05205	Proteoglycans in cancer	MMP2/VAV3/FLNB/HBEGF/RAC1/PPP1CB/ESR1/ERBB2/CCND1/MDM2	7.63E-04
hsa04380	Osteoclast differentiation	IFNGR1/BTK/RAC1/MAPK9/NCF2/Table1/IKBKG/FCGR2A	7.94E-04
hsa05212	Pancreatic cancer	RAC1/E2F1/MAPK9/ERBB2/CCND1/IKBKG	2.03E-03

## Data Availability

The data presented in this study are available on request from the corresponding author.
